The article "Impact of Helicobacter pylori Infection and Outcome of Anti-Helicobacter pylori Therapy in Patients with Reflux Laryngopharyngitis" was published in 2022. Journal: Evid Based Complement Alternat Med.

# Impact of *Helicobacter pylori* Infection and Outcome of Anti-*Helicobacter pylori* Therapy in Patients with Reflux Laryngopharyngitis

**DOI:** 10.1155/2022/8266321

**Published:** 2022-07-05

**Authors:** Huili Shen, Yijie Chen, Xiaohui Li, Jing Yan, Junjie Zhao, Demin Kong, Yanxia Shi, Zhihui Li, Jihong Wang, Na Shao, Zhenghui Wang

**Affiliations:** ^1^Department of Otolaryngology-Head and Neck Surgery, The Second Affiliated Hospital of Xi'an Jiaotong University, Xi'an, China; ^2^Department of Otolaryngology-Head and Neck Surgery, The Fourth People's Hospital of Shaanxi Province, Xi'an, China; ^3^College of Medicine, Xi'an Jiaotong University, Xi'an, China

## Abstract

**Objectives:**

This study was designed to explore the relationship between *Helicobacter pylori* (Hp) infection and reflux laryngopharyngitis (RLP) and to evaluate the outcome of anti-Hp therapy in improving RLP symptoms.

**Methods:**

A total of 410 patients with RLP were enrolled and tested for Hp infection. The association of Hp infection with reflux symptom index (RSI) and reflux finding score (RFS) was determined. Hp-positive patients received either a proton pump inhibitor (PPI) omeprazole alone (control group) or a combination regimen (experimental group) consisting of omeprazole, mosapride citrate, amoxicillin, and clarithromycin. Therapeutic outcomes were compared 4 weeks later.

**Results:**

Of the 410 participants, 290 were Hp-positive and 120 Hp-negative. Both RSI and RFS were significantly higher in Hp-positive patients than in Hp-negative patients. Hp infection status was positively correlated with RSI (*P* < 0.05) and RFS (*P* < 0.05). The overall response rate was higher in the experimental group than in the control group. Both the groups had a significant reduction in RSI and RFS after therapy, with a greater improvement in the experimental group (*P* < 0.05).

**Conclusion:**

Our findings establish a link between Hp infection and RLP. Anti-Hp therapy improves RSI and RFS in RLP patients. Therefore, Hp eradication drugs may be added to the PPI-based regimen in the treatment of RLP.

## 1. Introduction

Reflux pharyngitis (RLP), also known as laryngopharyngeal reflux disease, is characterised by inflammatory damage to the tissues of the upper aerodigestive tract caused by reflux of gastric contents [1]. Common symptoms include throat clearing, voice quality alteration, and globus pharyngeus. Although RLP has an adverse impact on the life quality of patients, its pathogenesis is still unclear. Moreover, there were no standard diagnostic and therapeutic methods available for RLP [2, 3]. For a long time in the past, reflux pharyngitis was often considered an extra-oesophageal manifestation of reflux gastro-oesophagitis, but now more and more scholars agree that these are two relatively independent diseases [4]. Reflux pharyngitis is characterised by acid reflux and heartburn in the stomach, with a higher incidence when lying down. Patients are associated with abnormal oesophageal peristalsis and prolonged exposure to gastric acid, with a daily repetition rate of up to 50 times and more [5]. Gastric manifestations such as acid reflux and heartburn are generally not present in reflux pharyngitis. Patients have only pharyngeal symptoms, which tend to occur in the upright position and are considered abnormal if they exceed four times per day [6].

The article "Impact of Helicobacter pylori Infection and Outcome of Anti-Helicobacter pylori Therapy in Patients with Reflux Laryngopharyngitis" was published in 2022. Journal: Evid Based Complement Alternat Med.

*Helicobacter pylori* (Hp) is a pathogenic bacterium that inhabits the gastric mucosa of humans. Hp infection has been suggested as an important etiological factor for gastroesophageal reflux diseases [7]. Clinically, the main drugs taken to treat HP are antibiotics (e.g., clarithromycin and amoxicillin), drugs to inhibit gastric acid secretion (e.g., omeprazole), and drugs to protect the gastric mucosa (e.g., bismuth potassium citrate), and triple therapy or quadruple therapy to kill *H. pylori* [6, 8, 9]. *H. pylori* is contagious and can be transmitted through food and utensils. Patients must develop good hygiene habits in daily life, wash their hands regularly before and after meals, and eat clean food, and disinfect utensils regularly can effectively kill *H. pylori* in their lives [10].

However, the relationship between Hp infection and RLP is still unclear. In the present study, we retrospectively analysed clinical data of RLP patients admitted in our hospital and assessed the association of Hp infection status and RLP. We also explored the outcomes of Hp therapy in patients with RLP.

## 2. Materials and Methods

### 2.1. General Information

A total of 410 patients diagnosed with RLP between August 2015 and August 2019 were recruited for retrospective analysis. Patients with Hp-positive RLP were sequentially assigned equally to the control and experimental groups according to the different treatment modalities. The study was approved by the Ethics Committee of Xi'an Jiaotong University (Xi'an, China) (approval no.#19879). Written informed consent for the study was obtained from each patient.

### 2.2. Inclusion and Exclusion Criteria

Inclusion criteria: (1) duration of disease >1 month; (2) patient age ≥18 years; (3) Hp-positive RLP patients.

Exclusion criteria: (1) presence of laryngopharyngeal trauma or systemic disease; (2) treatment with Hp within 3 months prior to RLP diagnosis; (3) receipt of a proton pump inhibitor (PPI) within 1 month; (4) laryngopharyngeal tumour.

The article "Impact of Helicobacter pylori Infection and Outcome of Anti-Helicobacter pylori Therapy in Patients with Reflux Laryngopharyngitis" was published in 2022. Journal: Evid Based Complement Alternat Med.

### 2.3. Hp Detection

Hp infection was examined using the ^14^C urea breath test [11]. Briefly, all the participants took an urea ^14^C capsule on an empty stomach 15 min before tests. The ^14^C content in the gas blew out from the patients was recorded by a YH04E Hp detector. The ^14^C results (expressed in dmp) were defined as: ≤99 dmp, negative; 99< dpm ≤149, uncertain; dpm >149, positive; 149< dpm ≤499, “+”; 499< dpm ≤1499, “++”; 1499< dpm ≤2499, “+++”; dpm >249, “++++.”

### 2.4. Treatment Protocol

The patients in the control group received a daily oral dose of 40 mg of omeprazole (Changzhou Siyao Pharmaceutical co., Ltd., Changzhou, China). For those with severe reflux symptoms, domperidone was added to the treatment regimen.

The patients in the experimental group were treated with a combination of omeprazole (40 mg/day), mosapride citrate (15 mg/day), amoxicillin (1 g BID), and clarithromycin (500 mg BID). The treatment was continued for 4 weeks in both the groups [12]. All the patients were advised to follow recommended dietary guidelines: i.e., intake of a restricted amount of food and no consumption of alcohol, coffee, tea, soda beverage, chocolate, or peppermint. Eating food should be avoided 3 h before sleep.

### 2.5. Reflux Measurements

Reflux symptom index (RSI) [13, 14] is a 9-item patient questionnaire scoring system used to assess severity of reflux symptoms. The parameters tested included hoarseness or dysphonia, chronic cough, difficulty swallowing, excess laryngeal secretions, heartburn or regurgitation, difficulty breathing, constant throat clearing, throat pain, and foreign-body sensation in the throat. Each item of RSI was scored from 0 (no symptom) to 5 (the most serious symptom). The total score of RSI was 45. Reflux finding score (RFS) [14, 15] is a 8-item clinical severity scale based on laryngoscopic findings. The parameters included subglottic edema, ventricular obliteration, mucosal hyperemia, vocal cord edema, laryngeal edema, posterior commissure hypertrophy, and thick endolaryngeal mucus. RFS scale ranges from 0 (no abnormal findings) to a maximum 26 (worst findings).

### 2.6. Therapeutic Outcome Assessment

Therapeutic outcome was graded as complete response (resolution of all symptoms in the throat and RSI ≤13), partial response (partial remission of symptoms, relief of mucosal hyperemia, edema, and hypertrophy, and RSI reduction but more than 13), and no response (no improvement in clinical symptoms, laryngoscopic findings, or RSI). The overall response rate (OR) was calculated using the formula of OR = (number of CR + number of PR)/145 × 100%, in which CR and PR means complete response and partial response, respectively.

The article "Impact of Helicobacter pylori Infection and Outcome of Anti-Helicobacter pylori Therapy in Patients with Reflux Laryngopharyngitis" was published in 2022. Journal: Evid Based Complement Alternat Med.

### 2.7. Statistical Analysis

Statistical analysis was performed using SPSS version 17.0. Differences in proportions were calculated using the chi-square test. The results expressed as mean ± standard deviation were compared using Student's *t*-test. Correlation analysis was determined using Pearson's correlation test. A level of *P* < 0.05 was significant.

## 3. Results

### 3.1. General Information

The control group had 80 males and 65 females, with a mean age of 55.6 ± 10.0 years (19–78 years). The experimental group also had 80 men and 65 women, with a mean age of 56.2 ± 11.9 years (22–80 years). There was no significant difference in clinicodemographic data of the 2 groups (*P* > 0.05).

### 3.2. Hp Detection Results

Of the 410 patients enrolled, 290 were Hp-positive and 120 Hp-negative (Table 1). No significant difference was noted between the Hp-positive and Hp-negative patients regarding gender (*P*=0.734) and age (*P*=0.366).

### 3.3. RSI and RFS Measurement Results

Table 2 shows comparisons of RSI and RFS between Hp-positive and Hp-negative patients. Of note, compared to Hp-negative patients, Hp-positive patients had a significantly higher RSI (32.66 ± 3.21 *vs*. 17.52 ± 2.53; *P* < 0.05) and RFS (21.68 ± 1.23 *vs*. 16.25 ± 1.04; *P* < 0.05).

### 3.4. Association of Hp Status with RSI and RFS

The Hp infection rate was positively associated with RSI (*r* = 0.770, *P* < 0.05) and RFS (*r* = 0.615, *P* < 0.05) in patients with RLP (Table 3), suggesting that Hp infection may be a risk factor of RLP.

### 3.5. Treatment Outcome Comparison

Hp treatment resulted in a significantly higher OR rate compared to the control group (90.34% vs. 74.48%, *P* < 0.05; Table 4). There was no significant difference in baseline RSI and RFS between the two groups before treatment (*P* > 0.05; Table 5). After treatment, RSI and RFS improved significantly in both groups. In addition, RSI and RFS were significantly lower in the Hp-treated group than in the control group (*P* < 0.05), indicating that patients derived better benefit from Hp treatment.

## 4. Discussion

RLP is a common laryngopharyngeal disorder that presents as an inflammatory injury to the upper aerodigestive tract. The incidence of RLP has increased in recent years, and this may be related to changes in dietary habits. It is estimated that over 50% of patients with voice abnormalities have reflux symptoms [16]. Multiple factors including oesophageal sphincter function, retention time of reflux contents, and pharyngeal mucosa susceptibility have an impact on the progression of RLP. Direct injury of pharyngeal mucosa by gastric reflux contents is regarded as an important cause of RLP [17]. RLP also involves vasovagal reflex-related injuries [18]. However, little is known about the exact pathogenesis of its RLP.

The article "Impact of Helicobacter pylori Infection and Outcome of Anti-Helicobacter pylori Therapy in Patients with Reflux Laryngopharyngitis" was published in 2022. Journal: Evid Based Complement Alternat Med.

Hp is a common pathogenic bacterium that lives in gastric mucosa. Accumulating evidence has linked Hp infection to gastric reflux diseases [19, 20]. Hp infection can cause excessive secretion of gastric acid, which can lead to abdominal distention, nausea, chronic gastritis, and gastric ulcers. In addition, Hp infection can cause oesophageal sphincter dysfunction and overproduction of acidic contents, which may exacerbate damage to the pharyngeal mucosa from acid reflux [21]. It has been reported that over 3 months of acid stimulation reduces the expression of E-cadherin and impairs the junction among laryngopharyngea mucosal cells, leading to submucosal muscle hypertrophy [22]. Another report suggests that Hp infection may contribute to the pathogenesis of RLP by altering the endocrine secretion of the gastric glands [23–25]. As a result of insufficient gastric acid, large amounts of undigested food are retained in the stomach, releasing spoiled gas and thus aggravating pharyngeal reflux [26–28].

It has also been confirmed that *H. pylori* prevents gastric acid production, which in turn can prevent reflux; that is, *H. pylori* infection is negatively associated with the development of a wide range of gastroesophageal reflux disease, contrary to the results of our study here [29, 30]. This occurs when the inflammatory infection of the stomach caused by *H. pylori* affects the entire gastric body, especially when it involves areas of gastric acid secretion [31]. The secretion of gastric acid is reduced because of the inhibitory effect of inflammatory cells on the mural cells [32]. Thus, in cases where *H. pylori* infection inhibits gastric acid secretion, *H. pylori* infection inhibits GERD episodes [33]. In some cases, however, the areas of the gastric body involved in gastric acid secretion are largely unaffected by *H. pylori* infection, so that gastric acid secretion is not reduced, but instead also leads to an increase in serum gastrin levels [34]. In this case, the risk of GERD associated with *H. pylori* infection is actually thought to be increased, which is consistent with the findings derived from our study.

In the present study, we show that Hp-positive RLP patients have a significantly higher RSI and RFS than Hp-negative RLP patients. There are positive correlations between Hp infection and RSI and RFS. The prevalence of Hp infection secondary to modification of dietary habits is emerging as a crucial factor of RLP progression. Therefore, we speculated that Hp eradication therapy may provide benefits in improving RLP symptoms. In our Hp-positive RLP patients, we compared the outcome of PPI and Hp therapies. It was found that anti-Hp therapy yields a significantly higher OR than PPI treatment (90.34% vs. 74.48%). Moreover, both RSI and RFS are improved to a greater extent in the experimental group than in the control group. Our results suggest the benefits of anti-Hp therapy in RLP patients.

The article "Impact of Helicobacter pylori Infection and Outcome of Anti-Helicobacter pylori Therapy in Patients with Reflux Laryngopharyngitis" was published in 2022. Journal: Evid Based Complement Alternat Med.

However, the limitations of the trial are clear, not least of which, Hp infection has not been assessed quantitatively, and we need a standard method of assessing treatment outcomes. We did not know the facts about the oesophageal status of these patients, so it was not clear if they had GERD, which was associated with RLP. Secondly, because this study was a retrospective analysis, the eradication rate was a missing number for us. Therefore, in a follow-up trial the investigators will be looking more closely at the response to eradication in HP-positive patients divided into eradicated and noneradicated patients. Finally, we consider that although ^14^C-UBT is proven to be safe, appropriate safety precautions must be taken for the storage, handling, and disposal of the radioactive test components. Our next step may be to choose the ^13^C isotope, as it is nonradioactive.

In summary, we indicate that Hp infection has a positive impact on RLP severity and progression. Compared to PPI treatment alone, Hp eradication therapy yields additional benefits in improving RSI and RFS in patients with RLP. These results warrant further studies in larger cohorts of patients with RLP.

## Figures and Tables

**Table 1:** *Helicobacter pylori* (Hp) detection results in 410 patients with reflux laryngopharyngitis.

Parameter	Hp infection status		*P* value
	Positive	Negative	
Gender			0.734
Male	160	64	
Female	130	56	
Age, years			0.366
≤35	28	16	
36–55	50	22	
56–75	124	55	
≥76	88	27	
Total	290	120	

**Table 2:** RSI and RFS in patients with or without *Helicobacter pylori* (Hp) infection.

Group	*n*	RSI	RFS
Hp-positive	290	32.66 ± 3.21	21.68 ± 1.23
Hp-negative	120	17.52 ± 2.53	16.25 ± 1.04
*P* value		<0.001	<0.001

RSI = reflux symptom index; RFS = reflux finding score.

**Table 3:** Association of *Helicobacter pylori* infection with RSI and RFS.

Parameter	*n*	*r*	*P* value
RSI	290	0.770	<0.001
RFS	120	0.615	<0.001

RSI = reflux symptom index; RFS = reflux finding score.

**Table 4:** Therapeutic outcome in the Hp therapy and control groups.

Group	*n*	CR (*n*, %)	PR (*n*, %)	NR (*n*, %)	OR (*n*, %)	*P* value^a^
Control	**145**	35 (24.14)	73 (50.34)	37 (25.52)	108 (74.48)	<0.001
Hp therapy	**145**	69 (47.59)	62 (42.76)	14 (9.66)	131 (90.34)	

CR = complete responses; Hp = *Helicobacter pylori*; NR = no response; OR = overall response; PR = partial response. ^*a*^*P* value was determined for the difference in OR between the control and experimental groups.

The article "Impact of Helicobacter pylori Infection and Outcome of Anti-Helicobacter pylori Therapy in Patients with Reflux Laryngopharyngitis" was published in 2022. Journal: Evid Based Complement Alternat Med.

**Table 5:** RSI and RFS before and after treatment.

Group	*n*	RSI		*P*	RFS		*P*
Control	**145**	32.67 ± 0.41	18.07 ± 1.05	≤0.001	21.66 ± 1.22	15.44 ± 0.54	<0.001
Hp therapy	**145**	32.65 ± 0.70	11.50 ± 1.73	≤0.001	21.72 ± 0.82	12.97 ± 1.50	<0.001
*P*		0.722	≤0.001		0.279	<0.001	

Hp = *Helicobacter pylori*.

## Data Availability

All data generated or analysed during this study are included in this published article.
